# Clinical Efficacy of Conventional Heparin Anticoagulation Combined with Apixaban in the Treatment of Patients with Cerebral Venous Thrombosis and Its Effect on Serum D-Dimer and FIB Expression

**DOI:** 10.1155/2021/4979210

**Published:** 2021-12-31

**Authors:** Xiaohui Dong, Xiaohui Liu, Yanqing Liu, Lili Jiang, Huiping Zhang, Bofeng Liu

**Affiliations:** ^1^Department of Neurosurgery, The No. 2 Hospital of Baoding, Baoding, 071051 Hebei Province, China; ^2^Operating Room, The People's Hospital of Qingyuan District, Baoding, 071100 Hebei Province, China

## Abstract

**Objective:**

The aim of this study was to explore the clinical efficacy of conventional heparin anticoagulation in combination with apixaban in the treatment of patients with cerebral venous thrombosis (CVT) and its influence on serum D-dimer **(**D-D) and fibrinogen (FIB).

**Methods:**

One hundred and fifty-seven consecutive CVT patients admitted to our hospital from January 1, 2006, to December 31, 2013, were allocated into two groups according to the different treatment methods, of which 95 cases received standard anticoagulation therapy (standard group (SG)) and the remaining 62 cases were given apixaban therapy (research group (RG)). The curative effects and the changes of coagulation function during the treatment, as well as the incidence of adverse reactions, were analyzed in the two groups. The changes of D-D and FIB levels before treatment and at days 1, 4, and 7 posttreatment were detected.

**Results:**

In treatment efficacy, RG was superior to SG. No evident difference was observed in the incidence of adverse events or coagulation function between the two groups. At day 1 posttreatment, D-D level was increased largely in both SG and RG, but the increase was much more significant in RG. However, D-D level was decreased gradually with time in both groups, and the reduction was more notable in RG. The FIB level in SG declined gradually with time after treatment and was higher than that in RG at the same time point. In RG, FIB was decreased gradually at day 1 and day 4 posttreatment, and its level at day 7 posttreatment showed no difference compared with that at day 4 posttreatment. Spearman's analysis identified that the higher the D-D level or the lower the FIB level at day 1 posttreatment was, the better the treatment efficacy was. After seven-day treatment, the lower the level of D-D and FIB was, the better the therapeutic effect was. Logistic analysis indicated that age, time of diagnosis, deep vein thrombosis (DVT), Glasgow Coma Scale (GCS) score, infection, Apixaban, D-D, and FIB all independently affect the treatment effect of patients.

**Conclusions:**

The combined use of Apixaban with heparin is high-performing and safe in the treatment of CVT. The changes of D-D and FIB levels during the treatment are strongly linked to the therapeutic effect, which can be used as plausible evaluation indexes for the efficacy of CVT.

## 1. Introduction

Cerebral venous thrombosis (CVT), also known as cerebral venous sinus thrombosis (CVST), has an annual incidence of approximately 1.32-1.57/100,000 people [1, 2]. It is a cerebrovascular disease with focal cerebral edema, venous cerebral infarction, epilepsy, and intracranial hypertension as the most prominent clinical characteristics, which often involves young adults and women of childbearing age and children [3, 4].

Although the mortality rate of CVT has been profoundly reduced with the improvement of treatment and diagnostic techniques, the mortality rate of severe CVT is still as high as 34.2% [5].

If CVT can be identified correctly at an early stage, patients could receive appropriate treatment in time, such as anticoagulation, intracranial pressure reduction, or neurosurgery. Thus, most patients diagnosed and treated at an early stage could have a favorable prognosis [6, 7]. After diagnosis by computed tomography (CT) or magnetic resonance (MR) venography, the standard treatment is to use heparin for anticoagulation first and then warfarin for anticoagulation [8]. It was reported that the treatment with anticoagulation for CVT was first demonstrated to be beneficial in a prospective study in 1991 [2]. The adoption of direct oral anticoagulants (DOAC), including dabigatran (a direct thrombin inhibitor) and the direct factor Xa (FXa) inhibitors such as apixaban, provides a viable alternative to vitamin K antagonists (VKA) or heparins for treating venous thrombosis and preventing stroke in atrial fibrillation patients in both the acute and longer-term phases. DOAC has been proved that it is more effective than VKA through more predictable pharmacokinetics, and it displayed similar efficacy to VKA in the treatment of acute venous thromboembolism (VTE), similarly, if not better, bleeding and mortality rates [1–6]. Subsequently, increased prescribing of these medications was shown in the last decade.

Apixaban belonged to an oral FXa inhibitor, which exerted an inhibitory effect on both free and clot-bound factor Xa, and also, it got approval in the clinical use of several thromboembolic disorders including reduction of stroke risk in nonvalvular atrial fibrillation, thromboprophylaxis following hip or knee replacement surgery, the treatment of deep vein thrombosis (DVT) or pulmonary embolism, and prevention of recurrent DVT and pulmonary embolism [4–6]. Apixaban was reported to be as effective as warfarin in the treatment of DVT and pulmonary embolism [9, 10]. More importantly, apixaban has many advantages including predictable pharmacokinetics and pharmacodynamics, low number of drug and food interactions, and relatively wide therapeutic window. However, only case reports and small sample studies have so far described the application of apixaban in CVT patients. Rao et al. [11] tracked a CVT patient who received apixaban in their study. During the follow-up, the patient had good tolerance to apixaban without any bleeding complications, and CT scan showed thrombolysis and recanalization, suggesting that apixaban may be a safe and viable method to treat CVT. Covut et al. [12] reported the therapeutic effect of apixaban on 5 CVT patients. Only 2 patients developed lower gastrointestinal bleeding 15 days after discharge. MR/CT venography showed that no patients had complete recanalization, 2 (40%) patients had partial recanalization, and 3 (60%) patients had no recanalization. During the treatment, no patients experienced clinically significant hemorrhage, nor did they experience thromboembolic events.

In this context, the therapeutic effect of apixaban in 62 CVT patients was analyzed, and the changes of D-dimer (D-D) and fibrinogen (FIB) levels in patients' peripheral blood were detected, so as to evaluate the therapeutic effect of Apixaban in this disease.

## 2. Materials and Methods

### 2.1. Study Participants

This study is a prospective cohort analysis, with 157 CVT patients admitted to our hospital between January 1, 2006, and December 31, 2013, and enrolled. The following are the inclusion criteria: all patients were diagnosed as CVT by X-ray and CT angiography and received oral anticoagulation therapy for at least 3 to 6 months. The following are the exclusion criteria: patients excluded were those (1) aged <18 years; (2) with severe liver and kidney dysfunction, mental abnormality, consciousness disorder, or inability to swallow oral drugs; (3) with CVT and central nervous system infection or severe head trauma; (4) with planned CVT surgical procedures; (5) with tumors; or (6) incomplete clinical data. This study conforms to the Declaration of Helsinki and has been ratified by the hospital's Medical Ethics Committee. All patients have signed the informed consent form.

### 2.2. Treatment Methods

Patients were divided into two groups based on different treatment methods. Of them, 95 patients were given standard anticoagulation therapy (standard group (SG)), and the other 62 patients were treated with apixaban therapy (research group (RG)). Standard treatment began with subcutaneous injection of low-molecular-weight enoxaparin (1 mg/kg) twice daily for 5-15 days. Warfarin was not used until the acute phase. In principle, warfarin and heparin were used repeatedly for 3-5 days, and heparin was withdrawn when the International Normalized Ratio (INR) of warfarin reached 2.0-3.0. The INR was detected regularly to adjust the dosage of warfarin, and the treatment duration was ≤24 weeks. After discontinuation of intravenous heparin therapy, apixaban was administered orally twice a day at a dose of 5 mg and measured 5 weeks later.

### 2.3. Follow-Up

After discharge, the patients were followed up by interview, which lasted for 6 months and was conducted once a month.

### 2.4. Outcome Measures

The following are the outcome measures:

1. Clinical efficacy: the efficacy was evaluated referring to the score standards of Clinical neurological impairment in Stroke Patients (1995).
2. Basically cured: the patients' functional impairment score reduced by 91-100%, and the degree of disability was grade 0.
3. Significantly improved: the patient's functional impairment score decreased by 46%-90%, and the degree of disability was 1-3.
4. Improved: the patient's functional impairment score decreased by 18%-45%.
5. No change: the patient's functional impairment score decreased by about 17%.
6. Deteriorated: the patient's functional impairment score decreased or increased by more than 18%.
7. Death: total effective rate = number of cases with (basically cured + significantly improved + improved)/total number of cases∗100%.
8. Statistics on adverse events: severe bleeding is defined as significant bleeding with a hemoglobin drop of more than 2 g/dL and/or requiring blood product infusion of more than 2 U, when the patient should stop the study medication.
9. Coagulation function analysis: the coagulation function, including activated partial thromboplastin time (APTT), partial prothrombin time (PT), and platelet (PLT), was compared between the two series before and after the last treatment.
10. Determination of D-D and FIB levels: fasting venous blood was collected before treatment and 1, 4, and 7 days after treatment for the determination of D-D and FIB via the SysmexCA7000 automatic blood coagulation analyzer (Hisenmeikang, Japan), specifically by immunoturbidimetry.

### 2.5. Statistical Analysis

SPSS19.0 was used for statistical analysis of the data. The counting data were represented by *n* (%), and the differences between groups were compared by a *χ*^2^ test. The measurement data were recorded as the mean ± SD. One-way ANOVA was used for comparison among groups, LSD test for back testing, repeated measures ANOVA for comparison at different time points, and LSD test for post hoc testing. Correlation analysis was done by Spearman's analysis, and the risk factors affecting efficacy were determined by logistic analysis. *P* < 0.05 was considered statistically significant.

## 3. Results

### 3.1. General Information

A total of 157 CVT patients were included in this study, including 95 cases in SG and 62 cases in RG. Basic data analysis revealed no statistical difference between RG and SG in terms of sex ratio, age, CVT diagnosis method, time of admission, time of diagnosis, hospitalization time, symptoms, DVT, GCS score, and infection (Table 1).

### 3.2. Therapeutic Effect Analysis

The total effective rate of patients in RG was higher than that in SG. RG had higher proportion of patients who were basically cured and lower proportion of patients who showed no change after treatment than SG (Table 2).

### 3.3. Adverse Event Analysis

Statistical analysis showed no difference in the incidence of single adverse event or total adverse event between the two series (Table 3).

### 3.4. Comparison of Coagulation Function between the Two Series

APTT, PT, and PLT identified no evident differences between the two series before and after treatment (*P* > 0.05) (Figure 1).

### 3.5. Changes of D-D and FIB Levels in the Two Series during Treatment

The pretreatment D-D and FIB levels showed no marked differences between the two series. On posttreatment day 1, D-D increased observably in both SG and RG, but the increase was more significant in RG. However, D-D decreased gradually with time in both series, and the reduction was more notable in RG. The FIB level in SG declined gradually with time after treatment and was higher than that in RG at the same time point. In RG, FIB decreased gradually on posttreatment day 1 and day 4, and its level at 7 days after treatment showed no difference compared with that at 4 days after treatment (Figure 2).

### 3.6. Correlation of D-D and FIB Levels with Therapeutic Effect

We analyzed the correlation of D-D and FIB with therapeutic effect one day and seven days after treatment. It was identified that the higher the D-D level or the lower the FIB level one day after treatment, the better the treatment effect. Seven days after treatment, the lower the levels of D-D and FIB, the better the therapeutic effect (Figure 3).

### 3.7. Analysis of Risk Factors Affecting Curative Effect

In order to analyze the factors influencing the curative effect of patients, we established a logistic model. The results identified that age, time of diagnosis, DVT, GCS score, infection, apixaban, D-D, and FIB can independently influence the curative effect of patients (Table 4).

## 4. Discussion

CVT is a rare cause of stroke, and the prognosis of patients is good. However, due to persistent neuropsychiatric symptoms and cognitive problems, approximately 1/4 of patients still cannot resume normal life and work [13, 14]. The current guidelines for the treatment of CVT are consistent, and anticoagulation is still the mainstay treatment method, with heparin or low-molecular-weight-heparin (LMWH) as the main drug [15, 16]. The optimal duration for anticoagulation treatment is usually 3 to 12 months. However, the condition of some severe CVT patients deteriorates after anticoagulation therapy [17], so the treatment strategy of CVT should be improved.

As an Xa inhibitor, apixaban has been approved in many countries for several indications [3–6]. The results of the key phase III clinical trials supporting its approval demonstrated that apixaban is an important alternative to existing anticoagulant therapies, such as VKAs or aspirin or LMWH, with an improved benefit-risk profile. Apixaban is an oral anticoagulant that can inhibit the production of thrombin by blocking the coagulation pathway both *in vivo* and *in vitro*. This paper analyzed the efficacy of apixaban in CVT patients on the basis of LMWH. The results exhibited that the patients supplemented with apixaban had better therapeutic effect. According to the score standards of clinical neurological impairment in stroke patients (1995), the basic recovery rate of patients treated with apixaban is 41.94%, which is notably higher than that of patients treated with LMWH (9.47%). Meanwhile, apixaban supplementation does not increase additional adverse reactions and has no significant effect on the coagulation function of the patients, suggesting that apixaban enjoys promising efficacy and safety in CVT treatment.

It is often applied to prevent thrombosis in cancer patients due to its merits in administration route, convenient use, and cost [18, 19]. Apixaban has been shown to reduce massive bleeding and VTE recurrence in the treatment of cancer-related venous thromboembolism (VTE) [20], as well as to prevent venous thrombosis and pulmonary embolism in the limbs of cancer patients [20, 21]. In the retrospective study of acute VTE, apixaban also showed no less efficacy and safety than rivaroxaban [22, 23]. However, in the current research on apixaban in treating CTV, the number of reported cases is small, although all of them show the positive effect of apixaban in treating CVT [11, 12]. Our research included 62 patients who received apixaban, which, to a certain extent, supplemented the evidence that apixaban actively treated CVT. We hope that more relevant studies will be conducted to provide a large number of case data.

The coagulation and fibrinolysis state were altered in CVT patients, and the changes play an important role in thrombolytic therapy [24, 25]. We analyzed the changes of D-D and FIB levels in CVT patients and found that the changes were closely linked to the treatment effect. The higher the D-D level in CVT patients one day after treatment, the better the curative effect; 7 days after treatment, the lower the D-D level of CVT patients, the better the curative effect, while the FIB level of CVT patients kept decreasing after treatment. D-D is a specific degradation product of cross-linked fibrin, and its increased level reflects secondary hyperfibrinolytic activity [26]. Higher D-D levels are found to be associated with thrombotic enlargement and acute attacks of symptoms. Although low D-D levels could not rule out CVT in patients with subacute or chronic diseases [27], D-D can be a reliable index for prognosis assessment and treatment guidance in patients with cerebral infarction [28, 29]. The final process of thrombus formation is the formation of soluble fibrin from FIB through the action of thrombin, and the content of FIB in the patient's body decreases. Generally speaking, FIB begins to decrease within 24 hours after thrombolytic therapy [30–32]. While there are currently few or even no reports on the correlation of D-D and FIB with treatment effect of CVT, more researches will be needed to provide more relevant evidence.

During CVT treatment, warfarin needs routine monitoring and dose adjustment, heparin requires intravenous administration, and there is a risk of heparin-induced thrombocytopenia. Apixaban has a high binding rate to plasma protein, and its metabolism depends on the liver and kidney, so it cannot be cleared through hemodialysis. Once uncontrollable bleeding occurs, it will be very dangerous. Hence, it is necessary to constantly detect the changes of physiological state of patients during medication. Though a randomized trial is undertaken, one thing is for sure: given the rarity of CVT, it will only succeed through collaboration of a large number of hospitals. Follow-up should be extended to observe the efficacy of them in CVT patients. More researches should be done to explore the underlying mechanism of apixaban/heparin or their combined use *in vivo*.

To sum up, apixaban combined with heparin is effective and safe in treating CVT, and the changes of D-D and FIB levels during treatment are closely related to the therapeutic effect, all indicating that their combined use can be valid evaluation indexes for the efficacy of CVT.

## Figures and Tables

**Figure 1:** Comparison of coagulation function between the two groups. (a) Comparison of PLT levels between the two groups before and after treatment. (b) Comparison of APTT levels between the two groups before and after treatment. (c) Comparison of PT levels between the two groups before and after treatment. APTT: activated partial thromboplastin time; PT: partial prothrombin time; PLT: platelet.

**Figure 2:** Changes of D-dimer and FIB levels in the two groups during treatment. (a) Changes in D-dimer levels. (b) Changes in FIB levels. ^∗^*P* < 0.05*vs.* standard group at the same time point; ^#^*P* < 0.05*vs.* before treatment; ^@^*P* < 0.05*vs.* one day after treatment; ^&^*P* < 0.05*vs.* four days after treatment. FIB: fibrinogen.

**Figure 3:** Correlation of D-dimer and FIB levels with therapeutic effect. (a) Relationship between D-dimer and therapeutic effect one day after treatment. (b) Relationship between D-dimer and therapeutic effect 7 days after treatment. (c) Relationship between FIB and therapeutic effect one day after treatment. (d) Relationship between FIB and therapeutic effect 7 days after treatment. FIB: fibrinogen.

**Table 1:** Comparison of clinical data between the two groups (*n* (%)).

	Standard group (*n* = 95)	Research group (*n* = 62)	*χ* ^2^/t	*P*
Gender			0.045	0.833
Male	43 (45.26)	27 (43.55)		
Female	52 (54.74)	35 (56.45)		
Age (years old)			2.860	0.582
<30	11 (11.58)	8 (12.90)		
30-39	25 (26.31)	10 (16.13)		
40-49	30 (31.58)	22 (35.48)		
50-59	14 (14.74)	13 (20.97)		
≥60	15 (15.79)	9 (14.52)		
Diagnostic method			3.502	0.321
CT combined with ductography	58 (61.05)	32 (51.61)		
MRI combined with ductography	24 (25.26)	24 (38.71)		
CT combined with CT venography	5 (5.26)	3 (4.84)		
MRI combined with MR venography	8 (8.42)	3 (4.84)		
Admission time (d)	4 ± 3	5 ± 4	1.786	0.076
Time of diagnosis (d)	7 ± 4	8 ± 5	1.386	0.168
Hospitalization time (d)	16 ± 8	17 ± 10	0.693	0.490
Symptoms			1.483	0.686
Aphasia	21 (22.11)	10 (16.13)		
Dyskinesia	28 (29.47)	23 (37.10)		
Mental disorder	16 (16.84)	9 (14.52)		
Intracranial hypertension	30 (31.53)	20 (32.26)		
Headache	88	39		
Deep vein thrombosis			0.209	0.648
Yes	10 (10.53)	8 (12.90)		
No	85 (89.47)	54 (87.10)		
GCS score			1.312	0.519
13-15	64	46		
9-12	18	11		
≤8	13	5		
Infection			2.026	0.155
Yes	17 (17.89)	6 (9.68)		
No	78 (82.11)	56 (90.32)		
C-reactive protein (mg/L)	10.25 ± 1.25	10.34 ± 1.36	0.215	0.830
Homocysteine (*μ*mol/L)	16.45 ± 1.55	16.50 ± 1.50	0.098	0.923
Drinking			0.993	0.319
Yes	49 (51.58)	37 (59.68)		
No	46 (48.42)	25 (40.32)		
Smoking			0.338	0.561
Yes	43 (45.26)	31 (50.00)		
No	52 (54.74)	31 (50.00)		

GCS: Glasgow Coma Scale; CT: computed tomography; MRI: magnetic resonance.

**Table 2:** Treatment effect analysis of patients in the two groups (*n* (%)).

	Standard group (*n* = 95)	Research group (*n* = 62)	*χ* ^2^	*P*
Basically cured	9 (9.47)	26 (41.94)	22.821	<0.001
Significantly improved	22 (23.16)	22 (35.48)	2.826	0.093
Improved	50 (52.63)	12 (19.35)	17.385	<0.001
No change	10 (10.53)	1 (1.61)	4.575	0.032
Deteriorated or dead	4 (4.21)	1 (1.61)	0.821	0.365
Total effective rate	81 (85.26)	60 (96.77)	5.431	0.020

**Table 3:** Adverse event analysis in the two groups.

	Standard group (*n* = 95)	Research group (*n* = 62)	*χ* ^2^	*P*
Recurrence	0 (0.00)	0 (0.00)	—	—
Intracranial hemorrhage	3 (3.16)	2 (3.23)	0.441	0.659
Gastrointestinal bleeding	2 (2.11)	1 (1.61)	0.376	0.707
Venous thrombosis	3 (3.16)	1 (1.61)	0.082	0.934
Thrombocytopenia	2 (2.11)	1 (1.61)	0.376	0.707
Abdominal discomfort	3 (3.16)	2 (3.23)	0.441	0.659
Elevated liver enzymes	1 (1.05)	0 (0.00)	Fisher	>0.999
Depression	7 (7.37)	5 (4.84)	0.113	0.737
Total incidence	21 (22.11)	12 (19.35)	0.171	0.679

**Table 4:** Logistic analysis of curative effect.

		Univariate		Multivariate	
		*P*	OR (95% CI)	*P*	OR (95% CI)
Gender	Male *vs.* female	0.561	1.358 (0.484-3.683)		
Age	<40 *vs.* ≥40 years	0.031	2.167 (1.072-4.381)	0.048	1.654 (1.014-2.716)
Hospitalization time (d)	Unclassified	0.124	2.023 (0.825-4.960)		
Time of diagnosis (d)	Unclassified	0.001	3.266 (1.644-6.475)	0.004	3.017 (1.426-6.316)
Hospitalization time (d)	Unclassified	0.039	1.036 (1.576-5.887)	0.382	1.688 (0.521-5.552)
Deep vein thrombosis	Yes *vs.* no	0.013	1.842 (1.152-2.977)	0.035	2.763 (1.093-5.388)
GCS score	>8 *vs.* ≤8	0.025	1.536 (0.284-1.987)	0.038	1.155 (0.653-2.118)
Infection	Yes *vs.* no	0.001	9.379 (6.482-13.166)	0.018	5.477 (1.247-23.318)
Drinking	Yes *vs.* no	0.034	2.158 (1.063-4.372)	0.739	1.227 (0.393-3.897)
Smoking	Yes *vs.* no	0.031	2.601 (1.068-6.269)	0.381	1.688 (0.531-5.552)
Complications	Yes *vs.* no	0.046	1.287 (0.739-2.286)	0.085	0.977 (0.188-1.964)
Treatment methods	Standard *vs.* apixaban	0.004	3.017 (1.426-6.318)	0.023	2.979 (1.185-7.648)
D-dimer	Unclassified	0.001	1.006 (1.664-5.411)	0.006	1.984 (1.232-3.264)
FIB	Unclassified	0.025	1.545 (0.284-1.979)	0.036	0.878 (0.394-1.194)

GCS: Glasgow Coma Scale; FIB: fibrinogen.

## Data Availability

All the raw data could be accessed by contacting the corresponding author if necessary.
